RETRACTED

# Circ-GTF2I/miR-590-5p Axis Aggravates Myocardial Ischemia-Reperfusion Injury by Regulating Kelch Repeat and BTB Domain-Containing Protein 7

**DOI:** 10.1155/2022/2327669

**Published:** 2022-05-27

**Authors:** Chunju Yuan, Jing Lu, Zhongpu Chen, Qianxing Zhou

**Affiliations:** Department of Cardiovascular Medicine, Zhongda Hospital Southeast University, Nanjing 210009, Jiangsu Province, China

## Abstract

**Purpose:**

We investigated the effect of the circular RNA (circRNA) general transcription factor IIi (GTF2I) on myocardial ischemia (MI) deterioration and neonatal rat cardiomyocyte damage.

**Methods:**

The cell experiment was performed by using neonatal rat cardiomyocytes. Moreover, a hypoxia/reoxygenation treatment model was established. Cell Counting Kit-8 assay was conducted, and EdU cell proliferation was detected. Cell apoptosis was detected *via* flow cytometry and quantitative RT-PCR (RT-qPCR). Binding detection was performed through a double-luciferase reporter assay. Interleukin-6 (IL-6), tumor necrosis factor-*α* (TNF-*α*), and lactate dehydrogenase (LDH) were detected *via* enzyme-linked immunosorbent assay (ELISA).

**Results:**

Compared with that in the sham and control groups, circ-GTF2I expression in MIRI and the hypoxia/reoxygenation treatment model was significantly upregulated *in vivo* and *in vitro*. The knockdown of circ-GTF2I relieved neonatal rat cardiomyocyte damage and MI. Further detection through the double-luciferase reporter assay confirmed that the binding site of circ-GTF2I to miR-590-5p and miR-590-5p was Kelch repeat and BTB domain-containing protein 7 (KBTBD7). ELISA and RT-qPCR results showed that circ-GTF2I induced the abnormal expressions of IL-6 TNF-*α*, LDH, Bax, Bcl-2, and Cyt-c in MIRI and the hypoxia/reoxygenation treatment models by regulating miR-590-5p and the heart development transcription factor KBTBD7.

**Conclusions:**

CircRNA circ-GTF2I aggravated MIRI and neonatal rat cardiomyocyte damage *in vivo* and *in vitro* by regulating miR-590-5p and the heart development transcription factor KBTBD7.

## 1. Introduction

Myocardial ischemia (MI) is the leading cause of death from cardiovascular diseases. The pathological basis of MIRI is insufficient myocardial blood supply caused by the reduction in coronary blood flow [1, 2]. Finding novel strategies and therapeutic targets, reducing cardiomyocyte damage and MI, and scientifically and rationally protecting the patient's heart function are common concerns of the medical community.

The circRNAs are a kind of single-stranded, closed RNAs formed by the reverse shearing of exons upon the maturation of precursor mRNAs [3]. Studies on MIRI and myocardial infarction have found a large number of miRNA-binding sites on circRNAs. Through specific binding to a certain sequence of the target miRNA *via* base complementation, a circRNA acts as a miRNA sponge and interferes with the function of a miRNA, therefore affecting the occurrence and development of cardiovascular diseases [4, 5]. A large number of studies have reported the potential of circRNAs as diagnostic markers. However, studies on the use of circRNAs as diagnostic markers in the cardiovascular field have not been widely reported. If circRNAs, an endogenous molecule, can be detected in the blood and their expression changes during MI, they are likely to be used as diagnostic markers for potential myocardial injury and will have considerable application prospects in the field of medical diagnosis and tissue engineering in the future. Mao et al. showed that circ-general transcription factor IIi (GTF2I) is upregulated in nerve injury [6]. However, the role of the circRNAcirc-GTF2I in MIRI and cardiomyocyte apoptosis has not been revealed. Therefore, we investigated the role of circ-GTF2I in MIRI.

RETRACTED

The miRNAs interact with complementary sequences in the 3′ nontranslation regions of protein-coding miRNAs to inhibit protein translation or cause mRNA degradation [7]. MiRNAs can adjust heart electric signaling conduction, myocardial contraction, cardiac growth, and cardiac function morphogenesis [8, 9]. However, the function of miR-590-5p, which is abundant in cardiomyocytes, has not been reported thus far.

The broad complex/tramtrack/bric-a-brac (BTB) protein family is a special transcription factor in eukaryotes that is closely related to the development of various multicellular organisms, including poxviruses, fruit flies, and vertebrates; its functions include transcriptional regulation, cytoskeleton regulation, tetramerization, ion channel gating, and protein ubiquitination and degradation [10]. Kelch repeat and BTB domain-containing protein 7 (KBTBD7), a transcription factor containing the BTB domain, has been proven to play an important regulatory role in heart development and cardiomyocyte differentiation, diversity, and morphogenesis [11, 12].

In this study, a bioinformatic database was used to predict that the intersection of regulatory circRNA in MIRI was circ-GTF2I and that the intersection of KBTBD7 expression in MIRI was miRNA-590-5p. The correlation between the clinicopathological indicators of MIRI and the expression levels of circ-GTF2I, miR-590-5p, and KBTBD7 was further analyzed. In addition, cell biology and animal model experiments were conducted to study the expression and influence of circ-GTF2I in abnormal cell biological behaviors in MI and to determine its target genes and biological mechanism to provide a scientific basis and strategies for the prevention and control of cardiomyocyte damage and MIRI occurrence.

RETRACTED

## 2. Materials and Methods

### 2.1. Animal Experiment

A total of 40 male SD rats were purchased from Charles River Co., Ltd. and randomly divided into 4 groups: the sham group, the MIRI model group, the MIRI + Len-siNC group, and the MIRI + Len-si-circ-GTF2I group. The male SD rats in the sham group were anesthetized with sodium pentobarbital (30 mg/kg) and fixed on a rat plate. Anesthesia was maintained through the mask inhalation of 2% isoflurane and 0.8 L/min oxygen. After thoracotomy, a suture line was passed under the left anterior descending branch without ligation. After 30 min, the suture line was extracted, and the chest was closed. Myocardial tissues and sera were collected after 72 h. The male SD rats for the MIRI model group were successfully anesthetized and fixed on rat plates. After thoracotomy, the left anterior descending branch was ligated with sutures, which were loosened after 30 min. Myocardial tissues and sera were collected 72 h later. After successful anesthesia, the MIRI model rats for the MIRI + Len-siNC group were fixed on rat plates. After thoracotomy, Len-siNC vector lentivirus (lentiviral vector construction and virus purification were performed in accordance with the instructions provided by Transgen, China) was injected into the left ventricular muscle with a syringe at the titer of 100 *μ*L 10^10^ pfu/mL. Myocardial tissues and sera were collected 72 h later. The MIRI model rats allocated to the MIRI + Len-si-circ-GTF2I groups were fixed on the rat plate after successful anesthesia. After thoracotomy, the Len-si-circ-GTF2I vector lentivirus (lentiviral vector construction and virus purification were performed in accordance with the instructions provided by Transgen, China) was injected into the left ventricle muscle with a viral syringe at the titer of 100 *μ*L 10^10^ pfu/mL. Myocardial tissues and sera were collected 72 h later [13]. Animal experiments are approved by the ethics committees of Zhongda Hospital Southeast University (no. 2019–010).

3,5-Triphenyltetrazolium Chloride Staining.

The heart was removed and rinsed through injection with 0.9% sodium chloride. It was rapidly frozen at−20°C for 20 min. The atrium and right ventricle were removed. The heart was cut into tissue slices with a thickness of 2 mm from the apex to the bottom perpendicular to the long axis of the heart. The sections were placed in 1% 2,3,5-triphenyltetrazolium chloride (TTC) phosphoric acid buffer (pH 7.4) in a dark environment and then incubated in a 37°C constant-temperature water bath for 30 min. After removing the specimen, the noninfarct myocardium appeared brick red, whereas the infarct myocardium was pale.

RETRACTED

### 2.2. Len-Si-Circ-GTF2I Interference Sequence and Virus Packaging

A RNA interference target sequence was designed for the circ-GTF2I sequence. The double-stranded DNA of the target sequence was synthesized. The pGCL-GFP vector was ligated through HpaI and XhoI double enzyme digestion and transformed. Positive clones were selected for PCR identification and sequencing. The 293T cells were infected with pHelper1.0 and pHelper2.0 plasmids under the mediation of Lipofectamine 2000. Packaging produced lentiviruses with infective capability. The virus titer was calculated on the basis of the number of GFP cells in 293T cells.

### 2.3. Isolation and Purification of Neonatal Rat Cardiomyocytes

One-week-old SD rats were disinfected, and their hearts were collected and immediately placed into precooled D-Hank's buffer. The hearts were cut open and rinsed 3 times. The ventricular muscle was collected and cut into 1 mm^3^ tissue blocks. Then, 10 mL of calcium-and magnesium-free 0.1% trypsin solution was added. After stirring at 37°C for 10 min, the upper suspension was absorbed and removed. A total of 10 mL of trypsin solution was added to the tissue for digestion. The digested supernatant was absorbed, and 10 mL of MEM medium (Gibco, Carlsbad, CA, USA) containing 15% fetal bovine serum (FBS, Biological Industries, Israel) was added. The medium was centrifuged at 10°C for 5 min at a speed of 130 × g. Then, 10 mL of 0.1% trypsin solution was added to the tissue for digestion, which was repeated several times until the tissue fragments were digested and the cells were separated. After suspending the collected cells, the undigested tissues were removed through filtration with a 200-mesh stainless steel mesh and then cultured in a CO_2_ incubator for 2h. Fibroblasts were removed, and neonatal rat cardiomyocytes were purified by using a differential adherent [14].

### 2.4. Cell Culture

The neonatal rat cardiomyocytes were cultured in MEM basic medium supplemented with 10% FBS and 1% penicillin-streptomycin (100 *μ*g/mL) (Solarbio, China) in a 37°C incubator with a humidified 5% CO_2_ atmosphere.

### 2.5. Hypoxia/Reoxygenation Treatment Model

Neonatal rat cardiomyocytes were diluted into 6-well plates at the density of 5 × 10^4^ cells per well. The culture medium was replaced with a serum-free medium after 8 h. The serum-free and sugar-free culture medium was replaced with the low-oxygen workstation (less than 0.1% O_2_, 5% CO_2_) culture after 6 h, and the cell culture medium was completely replaced after 4 h; the follow-up experiment was then carried out [15].

RETRACTED

### 2.6. Cell Transfection

Plasmids were purchased from Jiangsu Biomics Co., Ltd. (Jiangsu, China). The neonatal rat cardiomyocytes were transfected with Lipo3000 (Boster, China) in accordance with the manufacturer's protocol. After 24–36 h, the cells were used to test transfection efficiency *via* quantitative RT-PCR (RT-qPCR).

### 2.7. Cell Counting Kit-8 Assay

The transfected cells were diluted into 96-well plates at a density of 5 × 10^3^ cells per well. Each well was subjected to the Cell Counting Kit-8 (CCK8) assay (Solarbio, China). The cells were incubated for 1 h in the dark in a 37°C incubator. Absorbance was recorded at 450 nm with a microplate reader. Cell viability and proliferation rates were calculated after the detection values were obtained.

### 2.8. EdU Assay

The transfected cells were diluted in 96-well plates at a density of 5 × 10^3^ cells per well. Cell proliferation was measured by using a BeyoClick™ EdU Cell Proliferation Kit with Alexa Fluor 647 (Beyotime, China). The fluorescence levels of cells were observed by using a confocal laser scanning microscope (Leica, Germany).

### 2.9. Flow Cytometry

The neonatal rat cardiomyocytes were collected, and cell density was adjusted to 1 × 10^6^ cells/mL. Then, the cells were washed with 1×PBS twice, and 5 × 10^5^ cells were collected through centrifugation. Next, the cells were resuspended in 500 *μ*L of binding buffer. A total of 5 *μ*L of Annexin V-FITC was added and mixed. Finally, 5 *μ*L of propidium iodide was added and mixed at room temperature and reacted for 15 min in the dark. Flow cytometry was used to detect and analyze the proportion of cell apoptosis. The above experiment was repeated 3 times, and data were recorded.

### 2.10. RT-qPCR

Total RNA was extracted by using a RNA Fast kit (Solarbio, China). A HiScript®II Reverse Kit (Vazyme, China) was used to perform cDNA synthesis. The qPCR assay was performed by using SYBR Green PCR Mix (Boster, China) on an IQ5 PCR System (Bio-Rad, USA). The reaction procedures were as follows: 94°C for 1 min, 94°C for 30 s, 55°C for30 s, and 72°C for 30 s for 40 cycles. The following primers were used: circ-GTF2I, forward: 5′-ACAGAATTCGCCACCATGCTGGCCGTCGGCTG-3′, reverse: 5′- ACAGGATCCTCTGGGGAAGAAGTAGTCTGTATTGCTGAT-3′, Bax, forward: 5′-CTTCCAAGCCCACCCCAACT-3′, reverse: 5′- GGCCTCCAGGACCTTCAGC-3′, Cyt-c, forward: 5′-CTCCTCTGCATTGCCATTGT-3′, reverse: 5′-TGTGGCTCGAGGTATTGTCA-3′, Bcl-2, forward: 5′-CGACAAGCCTCCCAGGTTCA-3′, reverse: 5′- GTGCCACCCAGCCAGCTATC-3′, KBTBD7, forward: 5′-AAAGGAAGGGGACTACCAAAGAAA-3′, reverse: 5′-CACCTCCTCCACATCATACACCTG-3′, miR-590-5p, forward: 5′-TAGCTTATCAGACTGATGTTG-3′, reverse: 5′-TCAACATCAGTCTGATAAGCT-3′, U6, forward: 5′-GCTTCGGCAGCAACATATAC-3′, reverse: 5′-AACGCTTCACGAATTTGCGT-3′, GAPDH, forward: 5′-TGAGACCTTCAACACCCCAG-3′, reverse: 5′- GCCATCTCTTGCTCGAAGTC-3′.

RETRACTED

Quantitative analysis was performed by comparing 2^−ΔΔCt^ values. The analysis was repeated 3 times for each set. The expression of KBTBD7 mRNA was corrected on the basis of GAPDH expression. U6 was used to correct miRNA expression results.

### 2.11. Construction of the Dual-Luciferase Reporter Gene Plasmid

The primers for PCR amplification were designed in accordance with the 3′UTR sequence of the KBTBD7 gene from NCBI. The 3′UTR sequence fragment was synthesized through PCR amplification with DNA as the template. Electrophoretic products were identified through agarose gel electrophoresis. The restriction enzymes EcoRI and NotI were used as double-enzyme carriers. The enzyme digestion system was treated at 37°C for approximately 1 h. Then, the products were recovered and purified in accordance with the instructions of the Gel-Spin DNA Extraction Kit. The purified DNA solution was obtained. The purified digestion products were ligated. The system was connected in a warm bath at 50°C for 20 min. Competent *Escherichia coli* DH5*α* cells were thawed at room temperature. A total of 100 *μ*L of the product cells was mixed with the bonding product. The culture was oscillated in a shaker at 37°C and 220 r/min for approximately 1 h. After the bacteria had returned to their normal growth state, they expressed the antibiotic resistance gene that was encoded by the plasmid. The remaining medium was aspirated and mixed. Then, 100 *μ*L of the culture was spread on the LB solid medium containing ampicillin. Bacterial fluid was taken for PCR identification. Positive clones were sequenced. Sequencing results were compared with the target gene sequence. The wild-type plasmid containing the target sequence was named KBTBD7-3′UTR-WT, and the mutated plasmid with the site-directed mutation was named KBTBD7-3′UTR-MUT.

### 2.12. Dual-Luciferase Reporter Assay

After 24–48 h of plasmid cotransfection, the medium was discarded and the cells were washed with 200 *μ*L of 1×PBS. Deionized water was used to dilute 5×PLB (lysates) to 1×. The dilution was placed at room temperature before use. A total of 50 **μ**L of diluted 1×PLB was added to each well. The plates were shaken on a shaker for 20–30 min. A total of 10 *μ*L of supernatant was added to each well of a 96-well microplate, and 100 *μ*L of luciferase assay A premixed reagent was added to measure the intensity of the luciferase reaction. After the measurement was completed, 150 *μ*L of the premixed stop reagent was added to each well and allowed to stand for 2–5 s. Then, data were measured to determine the intensity of the internal reference *Renilla* luciferase reaction. The ratio of the two sets of data was calculated.

RETRACTED

### 2.13. TUNEL Assay

The TUNEL assay was performed to evaluate apoptotic cells in cervical cancer tissues. First, the slices were digested with protease K and deparaffinized. Then, the slices were incubated with TdT at 37°C for 1 h. The slides were reacted in HRP-labeled streptavidin and then detected with the stable chromagen DAB. Finally, the slices were observed by using a confocal laser scanning microscope (Leica, Germany).

### 2.14. ELISA Assay

Rat serum samples were obtained by centrifuging collected serum at 1500 × g for 10 min. The samples were stored at−20°C for interleukin-6 (IL-6), tumor necrosis factor-*α* (TNF-*α*), and lactate dehydrogenase (LDH) analyses. ELISA kits were purchased from Thermo Fisher Scientific (Waltham, MA, USA). The test was performed in accordance with the manufacturer's instructions.

### 2.15. Statistical Analysis

The SPSS 22.0 and GraphPad Prism 7.0 were used for statistical analysis. All data were expressed as mean ± standard deviation, and all results were repeated at least three times. Unpaired Student's two-tailed *t*-test was used to analyze the differences between the 2 groups. For multiple groups, data were analyzed *via* one-way ANOVA by using Tukey's post hoc tests. *P* < 0.05 was considered as statistically significant.

## 3. Results

### 3.1. Circ-GTF2I Is Upregulated in the Rat MIRI Model

We detected the expressions of IL-6 and TNF*-α* through ELISA and the level of cell apoptosis through TUNEL staining to determine whether the MIRI model was successfully established. As shown in Figures 1(a)–1(c), the expressions of IL-6 and TNF-*α* in the MIRI model group were significantly increased compared with that in the sham group, and cell apoptosis was induced in numerous myocardial tissues. Therefore, we confirmed that the rat MIRI model had been successfully established. Furthermore, we detected circ-GTF2I expression in the rat sham and MIRI groups. Circ-GTF2I expression in the MIRI group was significantly upregulated compared with that in the sham group (Figure 1(d)). Moreover, neonatal rat cardiomyocytes were successfully isolated, and the hypoxia/reoxygenation cell model was established. Similarly, the expression level of circ-GTF2I in the hypoxia/reoxygenation cell model was significantly higher than that in the normal neonatal rat cardiomyocytes (Figure 1(e)).

Knockdown of circ-GTF2I relieves cardiomyocyte damage in the neonatal rat cardiomyocyte damage model.

RETRACTED

The function of circ-GTF2I in MI has not been reported yet. We successfully established the neonatal rat cardiomyocyte damage model *via* hypoxia/reoxygenation treatment to study the function of circ-GTF2I in neonatal rat cardiomyocytes and transfected si-NC and si-circ-GTF2I into the neonatal rat cardiomyocyte damage model. RT-qPCR results indicated that si-circ-GTF2I transfection significantly inhibited the expression of si-circ-GTF2I in the neonatal rat cardiomyocyte damage model relative to that in the si-NC group (Figure 2(a)). Next, cell viability was determined *via* the EdU cell proliferation assay. The results indicated that compared with those in the si-NC group, transfected cells in the neonatal rat cardiomyocyte damage model in the si-circ-GTF2I group had remarkably higher fluorescence level and cell viability (Figure 2(b)). Cell apoptosis was detected *via* flow cytometry and RT-qPCR. Fewer apoptosis cells were observed in the si-circ-GTF2I group than in the si-NC group (Figures 2(c) and 2(d)). At the same time, compared with those in the si-NC group, the expression of the proapoptotic factor Bax was significantly downregulated and that of the antiapoptotic factor Bcl-2 was upregulated in the si-circ-GTF2I group (Figures 2(e) and 2(f)). All of these data revealed that the knockdown of circ-GTF2I relieved neonatal rat cardiomyocyte damage, promoted neonatal rat cardiomyocyte proliferation, and inhibited neonatal rat cardiomyocyte apoptosis.

### 3.2. Knockdown of Circ-GTF2I Inhibits MIRI *In Vivo*

We infected the MIRI rats with lentivirus, which also knocked down the expression of circ-GTF2I, to ensure consistency between the *in vitro* and *in vivo* experiments. We detected the expressions of IL-6, LDH, and TNF-*α* through ELISA to determine whether the knockdown of circ-GTF2I inhibited MIRI in the rat models. Compared with that in the MIRI and MIRI + Len-siNC groups, the expressions of IL-6, LDH, and TNF-*α* in the MIRI + Len-si-circ-GTF2I group had significantly decreased and were close to that in the sham group (Figures 3(a)–3(c)). Next, we measured the ratio of MIRI and myocardial infarction in rats. Notably, compared with that in the MIRI and MIRI + Len-siNC groups, the ratio of MIRI and myocardial infarction in the rats in the MIRI + Len-si-circ-GTF2I group had significantly decreased (Figure 3(d)). We detected cell apoptosis through TUNEL staining and RT-qPCR assay and found fewer apoptotic cells in the MIRI + Len-si-circ-GTF2I group than in the MIRI and MIRI + Len-siNC groups (Figure 3(e)). Moreover, compared with those in the MIRI and MIRI + Len-siNC groups, the expression of the proapoptotic factor Bax was significantly downregulated and the expression of the antiapoptotic factor Bcl-2 was upregulated in the MIRI + Len-si-circ-GTF2I group (Figure 3(f) and 3(g)). We also detected the inhibitory effect of si-circ-GTF2I *in vivo*. Our results showed that the expression of circ-GTF2I was significantly decreased in the myocardium injected with the lentivirus (Figure 3(h). TTC staining was used to detect the myocardial infarction area. The results showed that knocking down circ-GTF2I reduced the size of myocardial infarction with MIRI injury (Figure S1).

RETRACTED

### 3.3. MiR-590-5p Is the Target Gene of Circ-GTF2I

We first analyzed miRNA binding by circ-GTF2I to further study the mechanism of circ-GTF2I in MI. Bioinformatic results showed that circ-GTF2I could combine with miR-590-5p (Figure 4(a)). The further detection of the luciferase reporter gene confirmed that circ-GTF2I was bound to miR-590-5p (Figure 4(b)). The double-luciferase reporter was used to confirm the relationship between circ-GTF2I and miR-590-5p. Relative luciferase activity in the miR-590-5p mimic-WT group had significantly decreased compared with that in the mimic NC-WT group. However, the relative luciferase activity of the mimic NC-MT reporter did not noticeably change in the miR-590-5p mimic group. Next, we tested the expression of miR-590-5p in the neonatal rat cardiomyocyte model *via* RT-qPCR. Comparison with the si-NC and vector-NC groups revealed that the downregulation of the expression of circ-GTF2I could significantly enhance the expression of miR-590-5p in the si-circ-GTF2I group, whereas the overexpression of circ-GTF2I could inhibit the expression of miR-590-5p in the vector-circ-GTF2I group (Figures 4(c) and 4(d)). The results for circ-GTF2I and miR-590-5p showed that their coexpression had a negative correlation. Moreover, miR-186-5p expression in the MIRI and hypoxia/reoxygenation treatment groups obviously decreased compared with that in the sham and control groups (Figures 4(e) and 4(f)). On the basis of these results, we further speculated that circ-GTF2I might promote MIRI development by inhibiting miR-590-5p expression *in vivo* and *in vitro*.

Overexpression of miR-590-5p reverses the damage caused by circ-GTF2I to neonatal rat cardiomyocytes.

We successfully transfected mimic NC, miR-590-5p mimics, vector NC, vector circ-GTF2I, circ-GTF2I + miR-NC, and circ-GTF2I + miR-590-5p into the hypoxia/reoxygenation treatment model to further study the mechanism of miR-590-5p in MI. The overexpression of miR-590-5p could be verified in the miR-590-5p mimic group. First, we determined cell viability *via* the CCK8 assay. The results indicated that the transfected cells of the neonatal rat cardiomyocyte damage model in the circ-GTF2I + miR-590-5p group had remarkably higher OD_450_ values than those in the vector circ-GTF2I and circ-GTF2I + miR-NC groups (Figure 5(a)). Cell apoptosis was detected through flow cytometry and RT-qPCR. Fewer apoptosis cells were observed in the circ-GTF2I + miR-590-5p group than in the vector circ-GTF2I and circ-GTF2I + miR-NC groups (Figure 5(b)). At the same time, compared with those in the vector circ-GTF2I and circ-GTF2I + miR-NC groups, the expression levels of the proapoptotic factor Bax and cell apoptosis biomarker Cyt-c were significantly downregulated and the expression of the antiapoptotic factor Bcl-2 was upregulated in the circ-GTF2I + miR-590-5p group (Figures 5(c)–5(e)). On the basis of these results, we confirmed that the overexpression of miR-590-5p reversed the damage of circ-GTF2I to neonatal rat cardiomyocytes.

RETRACTED

### 3.4. Heart Development Transcription Factor KBTBD7 Is the Target Gene of miR-590-5p

The binding and interaction between genes related to heart development and miRNA have rarely been reported in MIRI studies. We analyzed the binding of genes related to heart development to miR-590-5p to further study the mechanism of genes related to heart development and miRNA in the MIRI models. Bioinformatic results showed that KBTBD7 could combine with miR-590-5p (Figure 6(a)). Further detection by using the luciferase reporter gene confirmed that KBTBD7 was bound to miR-590-5p (Figure 6(b)). The experimental idea here is the same as that presented in a previous article. Furthermore, we were surprised to find that once miR-590-5p was overexpressed in the miR-590-5p mimic group, the expression of KBTBD7 was significantly inhibited compared with that in the mimic NC and inhibitor NC groups; however, once miR-590-5p was inhibited, the expression of KBTBD7 was significantly upregulated in the miR-590-5p inhibitor group (Figure 6(c) and Figure S2). The results for KBTBD7 and miR-590-5p showed that their coexpression had a negative correlation. These results were completely in line with our expectation that circ-GTF2I would promote the expression of KBTBD7 and exacerbate MIRI and neonatal rat cardiomyocyte damage *in vivo* and *in vitro (*Figures 6(d) and 6(e)).

Knockdown of KBTBD7 reverses the proapoptotic effect of circ-GTF2I on neonatal rat cardiomyocytes.

We successfully transfected vector NC, vector circ-GTF2I, vector circ-GTF2I + shNC, and vector circ-GTF2I + sh-KBTBD7 into the hypoxia/reoxygenation treatment model to further verify whether circ-GTF2I could promote the expression of KBTBD7 and thus exacerbate MI. We found that KBTBD7 was significantly upregulated in the vector circ-GTF2I group and downregulated in the vector circ-GTF2I + sh-KBTBD7 group (Figure 7(a)). The results indicated that compared with those in the vector NC and vector circ-GTF2I + shNC groups, transfected cells in the vector circ-GTF2I group had remarkably lower OD_450_ values, whereas those in the vector circ-GTF2I + sh-KBTBD7 had a higher OD_450_ value (Figure 7(b)). Cell apoptosis was detected *via* flow cytometry and RT-qPCR. Surprisingly, fewer apoptotic cells were observed in the circ-GTF2I + sh-KBTBD7 group than in the vector NC and vector circ-GTF2I + shNC groups (Figure 7(c)). At the same time, compared with those in the vector NC and vector circ-GTF2I + shNC groups, the expression levels of the proapoptotic factor Bax and cell apoptosis biomarker Cyt-c were significantly downregulated, whereas the expression of the antiapoptotic factor Bcl-2 was upregulated in the GTF2I + sh-KBTBD7 group (Figures 7(d)–7(f)). On the basis of these results, we confirmed that the knockdown of KBTBD7 reversed the proapoptotic effect of circ-GTF2I in neonatal rat cardiomyocytes under hypoxia/reoxygenation treatment. We present a schematic of the relationship among circ-GTF2I, miR-590-5p, and KBTBD7 in MIRI (Figure 7(g)).

RETRACTED

## 4. Discussion

The circRNAs have been shown to be either directly or indirectly involved in the development and progression of many diseases, notably those in the field of oncology [16]. However, research on circRNAs in the cardiovascular system remains scarce [17]. Cardiovascular experiments mainly rely on the isolation and culture of primary cells. These experimental procedures are complicated, and the success rate and yield of cell isolation are not stable, further increasing the difficulty of research on circRNAs in the cardiovascular system [18].

The miRNAs can participate in the regulation of energy metabolism, oxidative stress, and cell calcium overload; they also play an important role in the regulation of MIRI injury and apoptosis [19]. Competitive endogenous RNAs (ceRNAs) are one of the most popularly studied regulatory modes of lncRNAs and are a new mode of gene expression regulation [20]. The expression level of lncRNA or circRNA in cells directly affects the number of miRNAs that can be bound by the corresponding mRNA [21].

Inflammatory response and apoptosis are the classic patterns of programmed cell injury and death in the body. They play a vital role in normal organ development and tissue homeostasis. Inflammation and apoptosis are involved in myocardial cell injury and death in many heart diseases, such as MI, myocardial infarction, and congestive heart failure [22]. Studies have shown that the excessive inflammation and apoptosis of cardiomyocytes during MIRI are important factors causing ischemic injury [23]. Therefore, the degree of inflammation and apoptosis can be used as indicators of successful MIRI modeling. In this study, we found that the expression of circRNA circ-GTF2I in the MIRI model was significantly increased, suggesting that circ-GTF2I might enhance MI. By using bioinformatics screening, we successfully found that the specific target gene of circ-GTF2I was miR-590-5p. Then, our luciferase reporter gene experiment further confirmed that circ-GTF2I was combined with miR-590-5p. Furthermore, through RT-qPCR and flow cytometry, we discovered that the overexpression of miR-590-5p could effectively inhibit the transcriptional level of circ-GTF2I, whereas the KBTBD7 transcription factor was negatively regulated by miR-590-5p. In conclusion, circ-GTF2I could promote cardiomyocyte apoptosis and MI occurrence and positively promote the biological function of the KBTBD7 transcription factor. In addition, the coexpression of KBTBD7 and circ-GTF2I was positively correlated. At the same time, circ-GTF2I could act as a ceRNA of miR-590-5p by competitively binding with miR-590-5p to regulate the expression of KBTBD7. MiR-590-5p negatively regulated the KBTBD7 transcription factor, whereas, as found for the first time in a study on the effect of the circ-GTF2I on MI, circ-GTF2I could bind to miR-590-5p and indirectly regulate KBTBD7 transcription factor. Previous studies have found that circRNAs can inhibit the deterioration of MI [24], whereas we found opposite findings for circ-GTF2I.

RETRACTED

We discovered that circ-GTF2I could aggravate MIRI and myocardial infarction. The overexpression of miR-590-5p could effectively inhibit the transcription level of circ-GTF2I and reduce the expression of Bax and Cyt-c, inhibit cardiomyocyte apoptosis, alleviate MIRI and myocardial infarction, improve left cardiac function, and participate in myocardial protection. These pieces of information indicated that miR-590-5p could be used as a new treatment for MI, bringing good news to patients with MIRI.

Many transcription factors with heart-specific expression and a key role in cardiac morphogenesis and development have been identified. The KBTBD7 transcription factor may participate in several important signaling pathways in the development of the heart and jointly regulate the normal occurrence of cardiac morphology and the maintenance of the normal function of the heart or is intrinsically related to the pathogenic mechanism of heart diseases [25]. We are the first to find that the expression of the KBTBD7 transcription factor in the MIRI model was significantly increased, suggesting that KBTBD7 might be involved in the vital activities of MI. By using bioinformatic screening, we successfully determined that the specific target gene of miR-590-5p was KBTBD7. Then, through a luciferase reporter gene experiment, we further confirmed that the combination of miR-590-5p and KBTBD7 transcription factor and miR-590-5p could inhibit the expression of KBTBD7. Moreover, through RT-qPCR, ELISA, and flow cytometry, we found that the knockout or downregulation of KBTBD7 could significantly reduce the expression of Bax and Cyt-c, inhibit cardiomyocyte apoptosis, and alleviate MIRI and myocardial infarction. Our results provided a novel understanding of the effect of KBTBD7 transcription factor on cardiac development and function. To summarize, we found that the KBTBD7 transcription factor was involved in MIRI and myocardial injury. Our findings play an important role in promoting research on the treatment of MIRI. In addition, circ-GTF2I was found to be a potential biomarker for acute myocardial infarction. Our study also revealed that circ-GTF2I could be a potential target in the treatment of myocardial infarction. Thus, our study provides a reference for subsequent biotherapy or drug development.

RETRACTED

The limitation of this study is that the upstream regulation mechanism of circ-GTF2I and the downstream target genes of circGTF2ImiR-590-5p/KBTBD7 axis require further study. Although this study found that circ-GTF2I might play an important role in MI, a large number of studies are needed before the real clinical application of this circRNA.

## 5. Conclusions

The circRNA circ-GTF2I was upregulated in MIRI models and was related to poor prognosis in MIRI deterioration and neonatal rat cardiomyocyte damage. Circ-GTF2I promoted MIRI deterioration and induced the neonatal rat cardiomyocyte damage by targeting miR-590-5p and KBTBD7.

## Figures and Tables

**Figure 1:** Circ-GTF2I is upregulated in the rat MIRI model. (a) Detection of IL-6 expression in the rat sham and MIRI models. (b) Detection of TNF-*α* expression in the rat sham and MIRI models. (c) Cell apoptosis was detected by TUNEL staining in myocardial tissue. (d) Circ-GTF2I was upregulated in the rat MIRI model. (e) Circ-GTF2I was upregulated in neonatal rat cardiomyocyte hypoxia/reoxygenation treatment model N = 10. All data were expressed as mean ± standard deviation, ^*∗*^*P* < 0.05, ^*∗∗*^*P* <  0.05, and ^*∗∗∗*^*P* < 0.001vs. control. Figure 1(a) (B) C and (D) ^*∗*^*P* < 0.05, ^*∗∗*^*P* < 0.01 vs. sham. Figure 1(e), ^*∗∗*^*P* < 0.01 vs. control.

**Figure 2:** Knockdown of circ-GTF2I relieves the myocardial cell damage in neonatal rat cardiomyocyte damage model. (a) Detection of circ-GTF2I transfection efficiency in the neonatal rat cardiomyocyte hypoxia/reoxygenation treatment model. (b) Detection of cell proliferation in the neonatal rat cardiomyocyte hypoxia/reoxygenation treatment model. (c) Cell apoptosis of neonatal rat cardiomyocytes was detected by flow cytometry. (d) Statistical results of neonatal rat cardiomyocyte apoptosis. (e) Bax expression level was detected in the neonatal rat cardiomyocyte hypoxia/reoxygenation treatment model. (f) Bcl-2 expression level was detected in the neonatal rat cardiomyocyte hypoxia/reoxygenation treatment model. The error bars in all graphs represented SD, and each experiment was repeated three times. ^*∗*^*P* < 0.05, ^*∗∗*^*P* < 0.01, and ^*∗∗∗*^*P* < 0.001*vs.* si-NC.

RETRACTED

**Figure 3:** Knockdown of circ-GTF2I inhibits the MIRI *in vivo.* (a) Detection of IL-6 activity in rat serum. (b) Detection of LDH activity in rat serum. (c) Detection of TNF-*α* activity in rat serum. (d) Detection of myocardial function in the rat MIRI model. (e) Cell apoptosis was detected by TUNEL staining in myocardial tissue. (f) Bax expression level was detected in myocardial tissue. (g) Bcl-2 expression level was detected in myocardial tissue. (h) Circ-GTF2I expression level was detected in myocardial tissue. *N* = 10. All data were expressed as mean ± standard deviation, ^*∗*^*P* < 0.05, ^*∗∗*^*P* < 0.01, and ^*∗∗∗*^*P* < 0.001*vs.* sham.

**Figure 4:** Circ-GTF2I acts as ceRNA of miR-590-5p to promote the apoptosis of cardiomyocytes. (a) The binding site information of circ-GTF2I targeting to miR-590-5p. (b) Dual-luciferase report detected circ-GTF2I binding to miR-590-5p. ^*∗*^*P* < 0.05 vs. WT. (c) Transfection efficiency detection of circ-GTF2I. ^*∗*^*P* < 0.05 vs. control. (d) MiR-590-5p expression level was detected the in circ-GTF2I knockdown model. ^*∗∗∗*^*P* < 0.001 vs. control. (e) MiR-590-5p expression level was detected in the rat MIRI model. ^*∗∗∗*^*P* < 0.001 vs. sham. (f) MiR-590-5p expression level was detected in the neonatal rat cardiomyocyte hypoxia/reoxygenation treatment model. ^*∗∗*^*P* < 0.01*vs.* control. Each experiment was repeated three times. All data were expressed as mean ± standard deviation.

**Figure 5:** The overexpression of miR-590-5p reverses the damage of circ-GTF2I to neonatal rat cardiomyocytes. (a) Detection of cell proliferation in the neonatal rat cardiomyocyte hypoxia/reoxygenation treatment model. ^*∗∗*^*P* < 0.01 vs. NC. (b) Cell apoptosis of neonatal rat cardiomyocytes was detected by flow cytometry. (c) Bax expression level was detected in the neonatal rat cardiomyocyte hypoxia/reoxygenation treatment model. (d) Cyt-c expression level was detected in the neonatal rat cardiomyocyte hypoxia/reoxygenation treatment model. (e) Bcl-2 expression level was detected in the neonatal rat cardiomyocyte hypoxia/reoxygenation treatment model. Each experiment was repeated three times. All data were expressed as mean ± standard deviation, ^*∗*^*P* < 0.05, ^*∗∗*^*P* < 0.01, and ^*∗∗∗*^*P* < 0.001*vs.* control.

RETRACTED

**Figure 6:** KBTBD7 is the target gene mediating the apoptosis regulation of miR-590-5p. (a) The binding site information of KBTBD7 targeting to miR-590-5p. (b) Dual-luciferase report detected KBTBD7 binding to miR-590-5p. (c) KBTBD7 expression level was detected in the miR-590-5p knockdown model. (d) KBTBD7 expression level was detected in circ-GTF2I overexpression model. (e) KBTBD7 expression level was detected in the rat MIRI model. ^*∗∗*^*P* < 0.01vs. sham. Each experiment was repeated three times. All data were expressed as mean ± standard deviation, ^*∗*^*P* < 0.05, ^*∗∗*^*P* < 0.01, and ^*∗∗∗*^*P* < 0.001vs. control.

**Figure 7:** The knockdown of KBTBD7 reverses the proapoptotic effect of circ-GTF2I on neonatal rat cardiomyocytes. (a) KBTBD7 expression level was detected in the neonatal rat cardiomyocyte hypoxia/reoxygenation treatment model. (b) Detection of cell proliferation in the neonatal rat cardiomyocyte hypoxia/reoxygenation treatment model. (c) Cell apoptosis of neonatal rat cardiomyocytes was detected by flow cytometry. (d) Bax expression level was detected in the neonatal rat cardiomyocyte hypoxia/reoxygenation treatment model. (e) Cyt-c expression level was detected in the neonatal rat cardiomyocyte hypoxia/reoxygenation treatment model. (f) Bcl-2 expression level was detected in the neonatal rat cardiomyocyte hypoxia/reoxygenation treatment model. (g) The schema of the relationship of circ-GTF2I, miR-590-5p, and KBTBD7 in MI. Each experiment was repeated three times. All data were expressed as mean ± standard deviation, ^*∗*^*P* < 0.05, ^*∗∗*^*P* < 0.01, and ^*∗∗∗*^*P* < 0.001 vs. control.

## Data Availability

The analyzed datasets generated during the study are available from the corresponding author on reasonable request.

## Supplementary Materials

Supplementary Materials Figure S1: The 2,3,5-triphenyltetrazolium chloride (TTC) staining was used to detect the myocardial infarction area. Figure S2: The expression of KBTBD7 was detected by Western blot.
